RETRACTED

# Pets at work: integrating pet-friendly initiatives into human resources for enhanced workplace harmony

**DOI:** 10.1186/s40359-024-01854-y

**Published:** 2024-07-02

**Authors:** Ana Junça-Silva, Marisa Galrito

**Affiliations:** 1 Instituto Universitário de Lisboa (ISCTE-IUL), Lisboa, Portugal; 2 Business Research Unit – BRU (UNIDE-IUL), Lisboa, Portugal

**Keywords:** Pet-friendly practices, Pets at work, Well-being, Work engagement, Basic psychological needs

## Abstract

**Aims:**

The representation of companion animals, or pets, has been changing recently. Research concerning how pets influence employees’ work-related well-being has also started to take its first steps. This research aimed to analyze (1) how managers perceive pet-friendly practices and their main effects at work, and (2) the impact of such practices on employees’ well-being and work engagement. Relying on the social exchange perspective and the self-determination theory it was hypothesized that pet-friendly practices would positively influence employees’ well-being and work engagement by satisfying their three basic needs (autonomy, competence, and relatedness).

**Methodology:**

Two studies with mixed methods were conducted. The first and exploratory study resorted to semi-structured interviews with six managers. The second was a two-wave study conducted with a large sample of workers (*N* = 379).

**Results:**

The first study highlighted the primary advantages and disadvantages of pet-friendly practices, along with the various obstacles and limitations, and proposed managerial strategies to overcome them. Managers generally expressed interest and enthusiasm about the topic but also pointed out challenges in implementing a pet-friendly strategy due to the limited number of empirical studies demonstrating its benefits. The second study’s findings indicated that pet-friendly practices positively impacted employees' work engagement and well-being by fulfilling their needs for competence, autonomy, and relatedness.

**Originality:**

Overall, Portugal is seen as having a conservative culture, which slows the dissemination and implementation of these measures. To overcome these challenges, several managerial recommendations have been proposed. Raising awareness and fostering discussion on the topic are crucial steps toward integrating pet-friendly policies into human resources management.

## Introduction

Recently, there has been growing interest in issues related to human-animal bonds [1]. In light of the role of companion animals, or pets, in modern society and the strong relationship between humans and their pets [2], understanding how they influence work-related life has been a recent concern for researchers and managers [3, 4]. For instance, some organizations are beginning to recognize the benefits of pets and their integration into work-related daily life [3]. These organizations have implemented pet-friendly practices—policies aimed at enhancing employee motivation and strengthening the bond between employees and their pets. Pet-friendly practices can range from simple or low-commitment options, such as offering pet insurance and telework, to more complex or high-commitment practices, like allowing employees to bring their pets to work. These initiatives are increasingly viewed as strategies to improve employee productivity, well-being, and retention [4, 5]. Additional benefits include lower absenteeism rates [6], higher morale [7], increased productivity [8], stronger organizational commitment [9], and an improved perceived workplace climate [10–13].

RETRACTED

The social exchange theory provides insights into the positive effects of pet-friendly policies [14]. According to this theory, employees continuously evaluate the balance between their contributions to the organization and the benefits they receive in return. When employees feel that their organization shares their values and supports their identity, they are more likely to be dedicated to their work. Consequently, for individuals who are pet owners or value pet-friendly environments, the existence of such policies within their organization is likely to enhance their sense of connection and engagement.

Work engagement describes a state where employees are emotionally and motivationally invested in their tasks, demonstrating energy, dedication and absorption in their work [15]. For example, if an employee has an elderly pet requiring medical attention during the workday, their engagement with their tasks may increase if the organization accommodates teleworking, even in a hybrid capacity. This accommodation signals support from the organization, fostering a deeper connection to work. Moreover, the employee's overall satisfaction with life may also improve [16], as they can work in proximity to their pets without concerns, contributing to their happiness [17, 18]. Consequently, pet-friendly practices have the potential to enhance both work engagement and employee well-being.

Drawing from self-determination theory (SDT; 19), we posit that fulfilling the fundamental psychological needs of autonomy, competence, and relatedness serves as the underlying mechanism connecting pet-friendly practices with both well-being and work engagement. Autonomy refers to the desire for psychological freedom in activities [19], while competence reflects the need to feel capable in navigating one's environment. Relatedness involves the yearning for positive connections with others [20]. According to SDT, these psychological needs are crucial for nurturing and sustaining intrinsic motivation in work contexts [21]. Therefore, organizations that foster practices supporting these needs are more likely to evoke heightened interest and engagement from employees [19]. By embracing pet-friendly initiatives, organizations can effectively nurture the fulfillment of these fundamental psychological needs, thereby positively influencing both work engagement and well-being.

RETRACTED

Despite the burgeoning interest among scholars, research investigating the advantages of pet-friendly policies on employee outcomes, particularly work engagement, remains limited [3]. Moreover, the stance of managers regarding pet-friendly practices remains largely unexplored. Therefore, in response to the specific call for research by Kelemen et al. [3] on the convergence of pets and organizational dynamics, this study aimed to achieve two primary objectives: (1) to scrutinize managerial perceptions of pet-friendly practices and (2) to assess the influence of these practices on employees’ well-being and work engagement by examining the fulfillment of their psychological needs.

This study makes significant contributions both theoretically and practically. Theoretically, it enriches the social exchange perspective and the SDT by integrating pets as pertinent variables within these frameworks. By recognizing pet-friendly practices as potential drivers of employees’ work engagement and well-being within the SDT framework, this research expands our understanding of the advantages associated with implementing such practices and their impact on various personal and work-related outcomes.

On a practical level, this research underscores the potential benefits of pet-friendly practices, offering valuable insights for researchers, managers, and policymakers alike. For instance, the findings from this study can inform the development of empirically grounded strategies for implementing pet-friendly initiatives. Additionally, it highlights the efficacy of simpler practices, often overlooked and underappreciated, in fostering employees’ well-being and work engagement. Such insights can guide stakeholders in crafting policies and practices that not only support employees but also contribute to organizational success.

## Theoretical framework

### The benefits of pets

The number of pets has significantly increased worldwide, and many are now considered family members [22]. This trend may be attributed to changes in the family unit and the recognition that pets contribute to both physical and psychological well-being [23].

RETRACTED

Despite the numerous advantages of adopting a pet, it also involves increased responsibility and concern when individuals need to be separated from them for extended periods, leading to anxiety and stress [24, 25]. This is especially true for those who must commute to work daily, resulting in prolonged periods away from home [4, 8]. Additionally, the strong emotional bond with pets [24] means that being apart from them can negatively impact individuals' concentration and performance at work [12].

Owning a pet offers various advantages, such as improved quality of life [10]. Mellor et al. [26] emphasize that pets enhance psychological safety perceptions [27], act as natural therapists [28], and boost mood [29]. Dogs and cats, in particular, help reduce anxiety and depression, mitigate loneliness, promote physical activity and playfulness, and enhance cardiovascular health [29, 30]. The presence of a dog or cat is associated with reduced stress and anxiety due to increased production of dopamine and serotonin—neurotransmitters known for inducing pleasure and having calming effects [27]. This is primarily due to the affection and companionship pets provide, as noted by Lebid and Simonova [31], offering support in both favorable and challenging circumstances. Additionally, the routine of caring for pets imparts a comforting sensation that helps maintain focus and organize daily tasks.

Pets have significant positive effects on their owners' health. For instance, a study by the Australian Baker Medical Research Institute demonstrated a direct correlation between pet ownership and a reduced risk of developing heart disease [32]. The benefits of pet ownership also include enhanced survival rates after heart attacks, reduced loneliness, improved social and emotional support [33], and a buffering effect against stress and challenging situations [25]. In a study investigating cardiovascular stress reactivity during a stress task performed in the presence of a dog or a close friend, Barker et al. [33] found that dog owners had lower physiological stress indicators when their pets were present. Another study observed that couples with pets exhibited lower blood pressure and heart rate at rest, as well as reduced systolic blood pressure and heart rate during a mental stress task [34].

Further human-animal interactions have a wide range of benefits; as highlighted by Biswas [35], interacting with friendly pets addresses various physical and mental issues, reducing blood pressure and improving cardiovascular health. The release of endorphins from such interactions produces a calming effect, alleviating pain, reducing stress, and enhancing overall psychological well-being [36]. For example, petting a cat or dog's head can lower blood pressure and induce relaxation, balancing physical and emotional stress [37]. Even the simple act of watching fish swim in an aquarium can relax tense muscles and reduce stress [38]. Stroking a dog or cat not only lowers blood pressure and heart rate but also increases serotonin and dopamine levels, promoting relaxation and mindfulness [22, 35]. Spending time playing and interacting with a pet further elevates serotonin and dopamine levels, hormones associated with positive emotions and well-being [39]. Overall, it is clear that pets provide a wide range of benefits to their owners.

RETRACTED

### The intersection of pets and work-related life

Pets’ representation is changing, and their owners are valuing them in such a way that their emotional attachment to them is becoming stronger [13]. Adding to this, pets may be a positive presence and a personal resource for their owners while working [17] which may justify why pets are being valued for organizational purposes, and the increased number of organizations adopting pet-friendly practices [40]. Pet-friendly practices are quite vast (even though often misunderstood); these are practices aimed at motivating employees by strengthening the bond with their pets and enhancing both human and animal welfare as the motivational factor. Organizations can become pet-friendly by implementing measures, such as allowing employees to bring their pets to work, allowing a few days of mourning for the loss of a pet, pet-based performance rewards such as canine hotel vouchers, allowing the employee to take their pet to the vet or pet daycare assistance [41].

These initiatives yield advantages for employees, leading to increased satisfaction and motivation [4, 42]. Furthermore, adopting pet-friendly practices benefits the organization by enhancing employer branding [43], fostering stronger ties within the community, attracting new talents and loyal stakeholders, and improving talent retention [8]. Simultaneously, these practices contribute to the creation of healthier working environments for employees [44] and a family-oriented atmosphere [45, 46]. For instance, by accommodating pets, organizations promote positive effects for employees, since many consider their pets family members [13, 47]. Some benefits of bringing pets to work or teleworking relate to better-balancing work and personal life [5]. Working near their pets allows employees to avoid worrying about leaving them home alone all day, particularly if the pet is elderly, has special needs, or requires regular medication for conditions such as diabetes or heart disease [36, 47, 48].

RETRACTED

These benefits are also relevant for the organization. Employees who bring their pets to work or work from home will likely work late to finish tasks since they do not need to rush home to care for their pets [17]. Other benefits include lower absenteeism rates, higher productivity, and improved employee relations [11, 42]. Pet-friendly practices meet the needs of employees and their customers and deliver significant advantages to organizations [30]. The presence of pets can increase productivity [3], foster socialization, enhance creativity, and reduce sedentary behavior [49]. For pets, it eliminates long hours of being alone, which in turn reduces their owners' concerns during the day and helps them stay more engaged with their work [50]. Therefore, pet-friendly practices can positively impact both performance and well-being.

### The relationship between pet-friendly practices and well-being indicators

Subjective well-being has been identified as subjective happiness and comprises an affective component related to the frequency of positive and negative emotions, and a cognitive component involving life satisfaction [16]. From this definition, happier individuals experience more positive affect than negative affect and hold a positive overall judgment about their lives as a whole [16]. Work engagement serves as a well-being indicator, encompassing vigor (physical energy for work), dedication (positive affective state during work), and absorption (focus on tasks) [15].

The positive effects of pet-friendly practices on well-being indicators may be supported by two theories: the social exchange theory and the SDT. First, based on the social exchange theory, employees are more likely to align and feel connected with an organization whose attributes, values, and practices resonate with their personal values; further, they tend to feel in debt with an organization that actively promotes conditions for them to feel happier [51]. Hence, when pet owners work for pet-friendly organizations, they likely become more engaged and happier with their work as a form of retributing what the organization does for them [3, 5, 22].

Second, SDT suggests that the degree of self-motivation varies across behaviors, identifying two main types of motivation that form a spectrum from intrinsic to extrinsic motivation [19]. Intrinsic motivation, at one end of this spectrum, is characterized by engaging in activities for their inherent enjoyment. At the other end is extrinsic motivation, driven by external rewards or outcomes. Additionally, SDT distinguishes between acting to avoid guilt (introjection), pursuing a valuable goal (identification), and acting in a way that reflects one’s identity (integration). Intrinsic motivation, along with identification and integration, are considered autonomous forms of regulation, highlighting a high degree of autonomy. The theory differentiates these types of motivation and emphasizes that different motives have distinct catalysts, concomitants, and consequences, with intrinsic motivation being the most relevant. This is because intrinsic motivation drives human behavior through the attainment of three basic needs [52]: autonomy (the feeling of volition), competence (the sense of effectiveness), and relatedness (the sense of connection with others). Fulfilling these needs is essential for employees to thrive and engage in their work [12], while thwarting these needs diminishes motivation and well-being [19]. Consequently, individuals strive to fulfill these needs, and when successful, they achieve psychological growth (e.g., intrinsic motivation), integrity (e.g., internalization and assimilation of cultural practices), and well-being (e.g., life satisfaction and psychological health [52]), as well as experiences of vitality [53] and self-congruence [54].

RETRACTED

The need for relatedness is a basic human need crucial for well-being [20] encompassing the desire to have stable, satisfying, and positive relationships [19]. From this standpoint, pet owners are likely to feel their need for relatedness is met if organizations implement pet-friendly practices that support their bond with their pets. For instance, allowing employees to bring their pets to work or work from home can fulfill their need for relatedness by being near their pets, leading to increased levels of both well-being and work engagement.

The need for competence refers to an individual's desire to feel effective and capable in areas they consider important [19]. Studies have consistently shown that feeling competent not only boosts self-confidence but also enhances well-being [55]. Additionally, research has demonstrated that achieving relevant goals predicts well-being and work engagement [56]. Therefore, pet-friendly practices may help individuals focus and concentrate on their tasks, facilitating goal attainment, and in turn, enhancing well-being and work engagement.

The need for autonomy is the desire to have flexibility and freedom in the tasks to be performed [19]. When employees have autonomy, freedom, and flexibility on the job they are also happier and more satisfied with it [21, 57]. Further, by having autonomy on the job employees tend to be more motivated to pursue organizational goals, which will likely influence work engagement [58]. Thus, pet-friendly practices, such as, telework or flextime, promote autonomy which will likely support employees’ need for autonomy and, in turn, will likely predict work engagement and well-being.

RETRACTED

To facilitate effective functioning in social contexts and improve psychological health and well-being the needs for competence, relatedness, and autonomy are essential. The fundamental idea is that environmental factors such as job design, human resources practices, and management have an impact on workers' motivations and experiences as they predict a set of basic psychological needs.

We propose that satisfying one's needs not only holds intrinsic value but also significantly boosts work engagement and well-being. Deci and Ryan [19] argued that dedicating energy to work on organizations with similar values can foster a sense of personal significance, thereby encouraging employees to immerse themselves more fully in their tasks. This notion has been supported by empirical research demonstrating that individuals whose psychological needs are met tend to exhibit higher levels of vigor and immersion in their work [58]. Research has shown that autonomous motivation for being near pets during work time significantly boosts employees’ need for satisfaction and well-being [12]. Thus, pet-friendly practices will likely satisfy their employees' needs, motivating them to do their tasks and thus increasing their work engagement and well-being.

Therefore, based on the SDT and the social exchange theory, it is expected that pet-friendly practices, by promoting organizational support and meeting psychological needs (autonomy, competence, and relatedness), increase well-being and work engagement (see Fig. 1).

**Fig. 1:** The proposed conceptual model

#### H1

Pet-friendly practices positively influence work engagement through the satisfaction of (a) autonomy, (b) competence, and (c) relatedness needs.

#### H2

Pet-friendly practices positively influence well-being through the satisfaction of (a) autonomy, (b) competence, and (c) relatedness needs.

### Overview of studies

The present research was supported by a mixed methodology. The first study was exploratory and embraced a qualitative approach to explore managers’ perceptions of pet-friendly practices, their implementation, and the perceived consequences. The second study, a two-wave study, aimed to test the effect of pet-friendly practices on well-being indicators (i.e., well-being and work engagement) by adopting the perspective of SDT and the social exchange framework.

## Study 1 – Pawsitive workplace: exploring managers' perspectives on pet-friendly practices

### Method

#### Participants and procedure

The first study adopts an exploratory approach to understand managers’ perceptions of pet-friendly practices and their main effects in the workplace. Hence, managers were selected through a non-probabilistic convenience sampling method. Six semi-structured in-depth interviews were conducted with managers from six organizations, who willingly volunteered to participate in the study after the formal email invitation.

RETRACTED

Participants were managers and exclusively belonged to the HR department of the organizations and were also actively engaged in organizational human resources policymaking. Invitations to participate in this study were sent through emails to potential participants meeting the predefined criteria. These emails clarified the objectives of the study, as well as the importance of their participation in it. After agreeing to participate in the interview, anonymity was guaranteed. From the 18 emails, 6 agreed to participate (response rate = 33.3%).

The participants exhibited job tenures ranging from 3 to 20 years, and their experience in human resources policymaking spanned from 2 to 15 years. Participants were 50% female and were aged between 30 and 55.

#### Instrument: semi-structured interview

This data collection method, as advocated by Bell et al. [59], facilitates the acquisition of comprehensive information, aligning with the exploratory nature of the study and at the same time allows interviewees to express their opinions with freedom of time and words. The interviewee's discourse was, however, guided by the pre-defined questions to obtain the information necessary for the first study’s goals. To this end, the interview scripts were built based on the literature review about pet-friendly practices to understand managers’ perceptions of pet-friendly practices [1, 3–6, 8, 11–13, 27, 33].

The initial segment of the interview focused on gathering background information from the respondents. In contrast, the second section comprised four open-ended questions delving into managers’ perspectives on pet-friendly practices. These interviews were individually conducted by the researchers, with the timing tailored to each respondent's availability throughout the week. At the beginning of the interview, they were assured that the data would be treated confidentially, and permission to record the interview was also asked. In this study, we chose to record the interviews to avoid taking notes during the interview, which could create a distraction. The interviews were conducted between July and September 2023, via Zoom, to facilitate the availability of the interviewees. The interviews lasted an average of about 45 min (*SD* = 10.23).

Notably, before data collection, the content validity of the interview questions underwent scrutiny by three PhD in human resources management and one expert in qualitative research. During the interviews, participants were encouraged to freely discuss, elaborate, and provide examples related to the pre-determined questions.

RETRACTED

### Data analysis

Given the study's design, researchers conducted a thematic analysis of the data using MAXQDA software. The thematic approach to qualitative data analysis, as outlined by Braun and Clarke [60], is theoretically flexible, making it applicable across various research domains; it involves coding data to identify emerging themes or patterns within interview transcripts. This initial phase involved transcribing all interviews and inputting them into the software. Following Corbin and Strauss' [61] framework, the researchers engaged in a three-stage process, encompassing open coding, axial coding, and selective coding. The iterative process involved generating open codes, juxtaposing, comparing, and unifying them in the second stage, and organizing the resulting themes into broader categories [62].

The creation of codes was based on the literature review of pet-friendly practices [1, 3–6]. With these procedures, we intended to recognize meanings at the level of similarities and differences and identify a coherence that would allow us to organize the information provided by the participants. The grouping of the main ideas referred to in the answers originated a categorical tree about the benefits, disadvantages, and limitations of pet-friendly practices.

To ensure rigor and validity, various strategies were employed, including member checking, peer debriefing, bracketing, and audit trailing. Member checking involved instructors reviewing and examining extracted codes/themes and the researchers' interpretations. Additionally, 10% of codes/themes were sent to a second coder, an experienced human resource associate professor, yielding a Cohen's Kappa coefficient of 0.98 for inter-coder reliability. Confirmability was maintained through a two-week audit trial conducted by another researcher who held a PhD in human resources management. The dependability and transferability of findings were enhanced by providing a comprehensive description of the research context, participants, and data collection procedures to facilitate potential replication in other settings.

Regarding researchers' positionality, their personal experiences with pet-friendly practices and human resources management informed their understanding of the context. However, to uphold trustworthiness, efforts were made to set aside personal biases during data analysis, ensuring that the researchers acted as objective data collectors, analysts, and collaborators with interviewees.

RETRACTED

### Results

The analysis done through MAXQDA allowed us to obtain five categories: 1) pets’ representations; 2) pet-friendly practices; 3) benefits; 4) disadvantages and limitations of implementing the practices; and 5) potential solutions to the limitations.

#### Pets’ representations

On the first point (see Fig. 2), three managers mentioned that pets were seen as children and that they required a lot of costs (*N =* 3) and consequently concern, responsibility, and caretaking (e.g., *“Many people already see their pets as their children”*). Additionally, some managers beckoned to the reasons that led them to perceive pets as it was outlined earlier. For instance, they emphasized the strong relationship between humans and their pets which harmed the harmony due to the frustration and worry of being away from them for many hours (*N =* 2; e.g., “*We often do not want to go to the office because we are attached to our animals*”).

**Fig. 2:** The first category and corresponding codes: pets’ representation

#### Pet-friendly practices

Regarding the second point, nine practices were identified. The most mentioned one was expense allowances such as pet insurance, and vouchers for veterinarian and hotel purposes (*N =* 11) (Fig. 3). When questioned about the topic and the practices they were aware of, and which ones were implemented at their organization, they pointed out examples such as telework (*N =* 7), awareness campaigns (*N =* 6), day of mourning in case of pets’ death (*N =* 6), ‘pet day’ at work (*N =* 5), the adoption of an organizational mascot (*N =* 5) and pet-walks (in which employees were allowed to take their pets) (*N =* 4). Managers emphasized six times the practice of the day of mourning in case of the pets’ loss of a pet (e.g., "*One thing my organization allows is remote work, and this practice is helpful because it allows us to be closer to our pets (…) And about the day of mourning, I think it makes perfect sense because I consider that animals are almost like children. (…) I'm sure that if one day I lose him, I'll be very grateful to have that day off from work*”).

**Fig. 3:** The second category and corresponding codes: pet-friendly practices

#### Pet-friendly practices: benefits

Managers identified two major benefits, one related to work and organizational-related benefits and another related to personal benefits. When analyzing the dimension of work and organizational benefits, four sub-categories were identified, namely productivity (*N =* 11), work engagement (*N =* 3), employee retention (*N =* 2), and organizational identification (*N =* 1). For instance, managers reported that the implementation of these practices could improve the sense of identification with the organization’s values and ideas, employees’ involvement, and engagement. Further, managers emphasized that pet-friendly practices could promote employee retention because when employees feel happy at work, retention increases. It was also cited that pet-friendly practices contribute to work-life balance. Finally, managers considered, in general, that pet-friendly practices allowed employees to be closer to their pets by taking more breaks in the case of telework, which helped to relieve occupational stress. An example is: “*I had a friend who was going through a tough time and her pets were her comfort to get through this time; so, she couldn't stay away from them for long (…) our CEO ended up implementing some pet-friendly practices because he saw many benefits for employee productivity*”.

RETRACTED

Moreover, the dimension of personal-related benefits included five sub-categories, namely: increased happiness and well-being (*N =* 7), more positive affective reactions during the day (*N =* 5), working nearby their pets (*N =* 4), stress reduction (*N =* 3) and work-life balance (*N =* 1) (see Fig. 4).

**Fig. 4:** The third category and corresponding codes: pet-friendly practices’ benefits

#### Limitations

In the fourth category, 11 disadvantages of pet-friendly practices were identified. All managers mentioned disadvantages, agreeing that these measures were still little known and that their implementation presented several challenges, mainly due to the conservative mind of the Portuguese population (*N =* 5) and to people who do not like pets or do not have them and as such do not fully understand (*N =* 2; e.g., “"*I think that one of the biggest problems is skepticism. In Portugal, I think that the big fight we are going to have will be skepticism and resistance. We see these practices implemented in the US and Brazil, but here it seems that the ideas arrive later.*").

Following the most mentioned pet-friendly practice (“allowing pets in the workplace”), the most mentioned obstacles to implementing it were allergies and phobias (*N =* 7). All managers mentioned that besides the difficulty that may exist to implement these practices, these also had an associated cost that would impact the organizational budget, and not all organizations were financially prepared for this cost (*N =* 5; e.g., “*The only less positive point is the higher cost that we now have.*”).

This implementation would be easier if the organizational budget were higher, and managers were open to taking risks and testing these measures (e.g., “*We have some financial health that allowed us to work on these practices and execute what are our dreams*”).

RETRACTED

Another sub-category emerged regarding the perception of inequality towards people who cannot take advantage of pet-friendly practices because they do not have pets (*N =* 3; e.g., “*Normally, when we implement a practice, we want everybody to be able to benefit from it, and this is also a problem. We would have to identify the people who have pets”).*

Another limitation pointed out was the age factor (*N =* 4), as older people are not as empathetic to these practices and end up not being as receptive to their implementation in organizations, which may be related to their conservative mindset (e.g., *“I think mentality is also associated with the age factor. The younger generations are more sympathetic than the older ones. (…) The mentality is associated with the age group factor”).*

Finally, support from managers was also highlighted as another salient sub-category (*N =* 5). Managers who have the responsibility of the decision-making, if they are not aware of employees' problems, cannot find solutions. In this sense, managers who are more attentive and closer to employees have a better perception of their well-being and thus can act or implement measures to combat the issues (See Fig. 5 for a summary).

**Fig. 5:** The fourth category and corresponding codes: pet-friendly practices’ limitations

#### Potential solutions for the limitations

It was also asked which solutions they considered to exist to overcome the obstacles and problems mentioned earlier. Telework was highlighted as a way to allow people to be closer to their pets, and consequently decrease the concern of leaving them alone for many hours while working (*N =* 9). Besides this, it was stated that to fight the population's conservative mindset, one should invest in information dissemination and awareness campaigns (*N =* 4; e.g., "*I think it is important that the subject is talked about among employees in an informal context*").

Finally, regarding the implementation process, when they were asked how they would do or did it in the case of implementing these practices, they answered that first of all, it should be important to diagnose employees’ perception of the potential implementation of pet-friendly practices (*N =* 8). They emphasized that this initial diagnostic was important to avoid any kind of revolt and discomfort and to involve them in the process (see Fig. 6; e.g., “But *for that, there has to be a diagnosis through a questionnaire that we give to the employees*”).

**Fig. 6:** The fifth category and corresponding codes: solutions

### Brief summary of results

Overall, a total of five categories were obtained: pet representation, pet-friendly, benefits, limitations, and solutions. From these categories, 30 subcategories were created (see Fig. 7 for a summary of the categories and the main sub-categories identified).

RETRACTED

**Fig. 7:** List of categories, sub-categories, and examples

In the first category “pets’ representation”, three subcategories are identified in which their image as “children” is the most identified category. In the second category “pet-friendly practices”, nine subcategories are identified, and the most mentioned one is having help with expenses (such as vouchers for veterinarians and hotels). The category "benefits" includes two main dimensions, one related to organizational and another related to personal benefits. In the organizational benefits, the most identified one is productivity increases, and in the personal advantages, managers highlight that pet-friendly practices lead undoubtedly to happier employees. Potential limitations include a total of 11 subcategories, of which the most mentioned is the potential existence of employees with allergies and phobias (in the case of allowing the presence of pets in the workplace). Finally, in the "solutions" category, five subcategories are identified, and the most mentioned solution is remote work.

## Study 2—Creating pawsitive work environments: a self-determination approach to pet-friendly practices and workplace well-being

### Method

#### Participants and procedure

The convenience sample was composed of a total of 379 working adults, of which 95% were female, aged between 18 and 74 years (*M* = 42.22; *SD* = 12.04). Most participants were married or living in a nonmarital partnership (53.8%), 30.1% were single, 14% were divorced and 2.1% were widowed. Most participants (36.4%) had a bachelor's degree, followed by a master's degree (29.3%). Overall, 27.4% were working in a hybrid regime, 52.2% in a full face-to-face regime, and 8.4% were completely teleworking. All participants had pets (*M* = 2.4; *SD* = 2.35). Overall, 92.7% had dogs, followed by cats (30.9%).

Two waves of data were collected. In the first stage, 558 surveys were distributed incorporating measures of pet-friendly practices, basic psychological needs, and socio-demographic characteristics. In total, 448 responses were received, yielding a response rate of 80.2%. In the second stage, questionnaires to measure work engagement and well-being were sent to the 448 participants who answered the first survey. At this stage, 399 completed surveys were gathered, generating a response rate of 71.50%. However, only 379 valid responses were considered after excluding invalid surveys (completed in less than 2 min or perfunctory answers), with an overall response rate of 67.9%. According to a power analysis (effect size of 0.2, error probability of 0.05), this sample size was considered sufficient.

RETRACTED

The only criterion to participate in the study was having at least one pet. Participants were part of the researchers’ professional network and were asked to participate in a study about pet-friendly practices via email. They were thoroughly informed about the nature and study’s goal and the confidentiality and anonymity of the data was warranted. Adequate information was provided about the demands that the project would place on them in terms of time and activities required from the respondents, as well as disclosure of confidential information. Respondents were also informed that they were free to participate, to decline to participate, or to withdraw from the research at any time. Since the questionnaires were shared online (via email), the above-mentioned information was provided in the cover letter of the questionnaire. Precautionary measures were used to minimize potential common method bias (CMB) [63]. Further, the items were randomized, and attention was set to screening questions in the questionnaires. Data was collected between October to December 2023.

#### Measures

##### Pet-friendly practices (T1)

We used the nine examples of pet-friendly practices identified in the previous study (e.g., “remote work”, and “mourning days in case of death of the animal”). Participants responded with a binary answer to whether their organizations had or not that practice implemented (“*yes*” and “*no*”); (α = 0.89).

##### Basic psychological needs (T1)

We measured the three dimensions of psychological needs: autonomy, relatedness, and competence, based on work-related basic need satisfaction [64, 65]. It included two items per dimension: autonomy (e.g., “I feel I can pretty much be myself at work”), relatedness (e.g., “I feel people at work care about me”), and competence (e.g., “I feel competent and capable”). Participants rated on a five-point Likert scale ranging from “*not at all*” to “*extremely*”. The Cronbach's alpha ranged from 0.84 to 0.87.

##### Subjective well-being (T2)

Subjective well-being was measured with the short form of the satisfaction with life scale [66]. It included three items, such as “I feel that my life is getting closer to my ideals”. Participants rated it on a five-point Likert scale ranging from ‘*strongly disagree*’ (1) to ‘*strongly agree*’ (5); (α = 0.92).

##### Work engagement (T2)

Work engagement was assessed with the three-item Ultra-Short Work Engagement Scale [67] (e.g., “I have been feeling full of energy”). It was rated on a 5-point Likert scale that ranged from 1 – *never* to 5 – *always*; (α = 0.88).

RETRACTED

##### Control variables

We used participants' age as a control variable because it could account for influences on well-being and work engagement, as there have been identified differences in the way elders and younger experience affect and their subsequent levels of well-being [68, 69].

### Data analysis

In the proposed mediating model (see Fig. 1), there were three types of variables: (1) predictor (pet-friendly practices); (2) two criterion variables (i.e., work engagement and well-being); and (3) three mediators (basic psychological needs: competence, autonomy and relatedness). SPSS 28.0 and the software JASP (version 0.14.1) were used to test the proposed research models. First, descriptive analysis was conducted to calculate the mean and standard deviation for each variable. Second, correlational analyses were performed to examine whether pet-friendly practices were associated with the mediators and the criterion variables. Fourth, the measurement model’s goodness of fit was evaluated. In this regard, we found that the Root Mean Square Error of Approximation (RMSEA) < 0.08, Standardized Root Mean Squared Residual (SRMR) < 0.08, Comparative Fit Index (CFI) > 0.90, and Tucker-Lewis Index (TLI) > 0.90 evidenced a good fit [70].

### Results

#### Common method bias and multicollinearity issues

Although we have followed some recommended procedures to reduce the potential common method bias—i.e., using closed-ended questions mixed in the survey (e.g., “I like ice creams”) and resorting to previously validated surveys to assess the variables under study—it cannot be completely avoided [63]. Hence, to understand its presence in the study we followed some recommendations.

First, we performed Harman’s single-factor test to check for common method bias. The findings showed that the first factor only accounted for 35.91% of the total explained variance; hence, the common method bias was not a serious issue.

Second, as Kock suggested [71], we also performed a full collinearity evaluation test to check for the potential common method bias. The results demonstrated that all the variance inflation factor values ranged from 1.04 to 2.63; because the values were less than the cut-off point of 3.33, multicollinearity concern was not a severe issue in this study.

At last, we performed four confirmatory factor analyses (CFA) to confirm the independence of the variables under study. To assess the adequacy of the model and compare it with other reasonable alternative models, we analyzed diverse fit indices, namely CFI, TLI, SRMR, and RMSEA. Model 1 was the hypothesized six-factor model comprising separate scales for pet-friendly practices, competence, autonomy, relatedness needs, work engagement, and well-being. Model 2 was a three-factor model where work engagement and well-being were combined into a unique factor, plus the three psychological needs were loaded onto one factor and another one for pet-friendly practices. Model 3 was a two-factor model where work engagement, well-being, and the three psychological needs were combined into a single factor. Model 4 was a one-factor solution in which all items were loaded onto a single factor. Table 1 shows that the six-factor model (Model 1) provided the best fit for the data (χ2/d*f* = 1.51, *p* < 0.001, CFI = 0.99, TLI = 0.9, SRMR = 0.06, and RMSEA = 0.04 CI 95% [0.03, 0.05]) (see Fig. 8), and all other alternative models evidenced a poorer fit. These results together with the Cronbach alpha reliability scores across all the measurement scales evidenced the discriminant and convergent validity of the study; hence, we proceeded with the hypotheses testing.

RETRACTED

**Table 1:** Confirmatory factor analysis results (Study 2)

Models	χ2	df	CFI	TLI	RMSEA	SRMR
Model 1	235.500	155	0.99	0.99	0.04	0.06
Model 2	749.717	167	0.98	0.98	0.11	0.08
Model 3	1,520.475	169	0.97	0.97	0.16	0.11
Model 4	5,224.882	170	0.88	0.87	0.31	0.31

**Fig. 8:** Confirmatory factor analysis model plot (Study 2)

#### Descriptive statistics

Table 2 shows the descriptive statistics and correlations between the variables under study. All the variables showed significant associations between them, however, age was not significantly associated with the main variables. Further, composite reliability and AVE values for all variables were greater than the threshold values of 0.7 and 0.5, respectively. The ranges of skewness (from − 0.88 to 1.09) and kurtosis (from − 0.56 to 1.47) for all the main variables were in the acceptable range (-2 to + 2) to perform structural equation modelling.

**Table 2:** Descriptive statistics, correlations, and reliabilities

Variable	*M*	*SD*	1	2	3	4	5	6	7
1. PFP	1.51^1^	0.78	(0.89)						
2. Autonomy needs	3.82^1^	1.10	0.09	(0.86)					
3. Relatedness needs	3.95^1^	1.10	0.17**	0.62**	(0.87)				
4. Competence needs	3.78^1^	1.03	0.13*	0.71**	0.60**	(0.84)			
5. Work engagement	3.18^1^	1.04	0.19**	0.50**	0.57**	0.60**	(0.88)		
6. Well-being	3.26^1^	1.04	0.12*	0.40**	0.47**	0.44**	0.69**	(0.92)	
7. Age	42.11	12.04	0.07	0.01	-0.03	0.07	0.03	-0.04	
8. Sex	-	-	-0.03	0.105	0.08	0.08	0.13*	0.12*	

*Cronbach* alfas are in brackets

*PFP* Pet-friendly practices

*N =* 379; ^*^p < 0.05 ^**^ *p* < 0.001

^1^Scale ranging from 1 to 5

^2^Sex codes: 1 – female; 2 – male

#### Hypotheses testing

The structural equation model fitted the data well: *χ2*_(313)_ = 1.39, *df* = 35, *p* < 0.001, CFI = 0.99, TLI = 0.99, RMSEA = 0.04, 90% *CI* [0.09;0.16]), SRMR = 0.03. The standardized path coefficients among the variables are presented in Fig. 9.

RETRACTED

**Fig. 9:** The path estimates of the proposed mediation model (Study 2)

First, the tests of indirect effects indicated that the need for competence and relatedness significantly mediated the relationship between pet-friendly practices and work engagement (*β* = 0.06; *p* < 0.01; *95%CI* [0.02;0.13]; *β* = 0.03; *p* < 0.01; *95%CI* [0.03;0.13], respectively). The findings showed that the need for autonomy did not mediate the relationship between pet-friendly practices and work engagement (*β* = 0.01; *p* > 0.05; *95%CI* [-0.00; 0.05]). The overall model explained 44% of the variance in work engagement (*R*^2^ = 0.44) (Table 3). Hence, hypothesis 1a did not receive support; however, hypotheses 1b and 1c were supported by the data.

**Table 3:** The mediation model total, direct and indirect effects (Study 2)

Indirect effects					Estimate	*P*	CI 95% LLCI	ULCI
PFP	→	NEED_AUT	→	WE	0.003	0.57	-0.00	0.03
PFP	→	NEED_REL	→	WE	0.051**	0.001	0.02	0.10
PFP	→	NEED_COMP	→	WE	0.048*	0.02	0.01	0.11
PFP	→	NEED_AUT	→	Well-being	0.004	0.48	-0.00	0.03
PFP	→	NEED_REL	→	Well-being	0.050**	0.001	0.02	0.10
PFP	→	NEED_COMP	→	Well-being	0.027*	0.04	0.01	0.08
**Total indirect effects**								
PFP	→	Work engagement			0.102**	0.001	0.03	0.18
PFP	→	Well-being			0.082**	0.001	0.03	0.14
**Direct effects**								
PFP	→	Work engagement			0.086*	0.05	0.00	0.178
PFP	→	Well-being			0.042	0.40	-0.061	0.147
**Total effects**								
PFP	→	Work engagement			0.188**	< .001	0.09	0.31
PFP	→	Well-being			0.124*	0.02	0.02	0.25

*PFP* pet-friendly practices, *WE* Work engagement

*N =* 379; ^*^p < 0.05 ^**^ *p* < 0.001

Second, the results evidenced similar patterns for well-being. The need for autonomy did not mediate the relationship between pet-friendly practices and well-being (*β* = 0.01; *p* > 0.05; *95% CI* [-0.00; 0.05]). On the oppositive, the results showed that both psychological needs (competence and relatedness) mediated the relationship between pet-friendly practices and well-being (*β* = 0.04; *p* < 0.05; *95%CI* [0.01; 0.10]; *β* = 0.07; *p* < 0.01; *95%CI* [0.03; 0.14], respectively). The overall model explained 27% of the variance in work engagement (*R*^2^ = 0.27). Hence, while hypothesis 2a did not receive support, hypotheses 2b and 2c received support from the data.

## Overall discussion

The motivation behind this study stems from the scarcity of research exploring the impact of pet-friendly practices on both organizational and personal outcomes [3]. Furthermore, there remains a notable lack of pet-friendly organizations, many of which still lack sufficient knowledge about this topic. Given the significant role that pets play, it is imperative to investigate and understand the reasons for the limited research on pet-friendly organizations. Thus, this research responds to the call for more studies on how pet-friendly practices influence employees' outcomes, such as well-being and work engagement [3].

RETRACTED

Comprising an exploratory and a correlational study, this research identifies specific categories of pet-friendly practices that contribute to a harmonious workplace and promote employee well-being. Moreover, the second study employs a social exchange and self-determination perspective to examine whether pet-friendly practices can help employees fulfill their basic psychological needs, namely autonomy, relatedness, and competence. The findings suggest that satisfying these needs may subsequently enhance both work engagement and well-being levels.

Overall, the findings of the first study suggest that pet-friendly practices are relatively unfamiliar to managers. It seems they often associate such practices solely with allowing pets in organizational facilities. However, managers also acknowledge that despite Portugal’s conservative culture, pet-friendly practices could offer benefits to employees who own pets and have strong bonds with them.

The findings of the second study provide evidence of the positive impact of pet-friendly practices on both work engagement and well-being. This impact is attributed to the satisfaction of the needs for relatedness and competence.

### Theoretical implications

First, the findings from the first study show that although managers are familiar with pet-friendly practices, there are still many doubts and uncertainties about implementing them and their potential benefits. For them, pet-friendly practices are associated with taking the pet to the workplace and can contribute positively to several factors, namely productivity, reduced stress and anxiety, improved work engagement, and identification with the organization’s values, which is aligned with some studies in the field [1, 5, 18]. Indeed, a pet, considered a child to many people and a family member, who stays home alone during the workday can be a reason for deconcentrating and creating anxiety at work [41]. This is consistent with empirical findings. A study conducted by Rossbach and Wilson [72] showed that pets directly contribute to decreased absenteeism and turnover, increased productivity, and lower medical, legal, and insurance costs, which are all outcomes of interest to organizations. People are happier and more relaxed in the presence of a pet [3]. In a separate study, pet owners reported experiencing lower stress levels when they were near their pets during the day. Unlike typical working days, where they might feel increased stress and anxiety, these feelings were not as pronounced when they remained near their pets throughout the day, alleviating the need to rush home to attend to them [48]. The study concluded that, compared to their coworkers who did not have pets, pet owners who left their pets at home while they went to work experienced significantly higher levels of stress by the end of the day [33].

RETRACTED

Secondly, the results of the second study reveal that the need for autonomy does not act as a mediator in the relationship between pet-friendly practices and both work engagement and well-being. In other words, while pet-friendly practices positively impact work engagement and well-being, they do not do so through the need for autonomy. This could be attributed to the diverse range of pet-friendly practices measured by the instrument, spanning from pet insurance to telework or bringing pets to work. The inclusion of the different pet-friendly practices may have biased the mediating model. Furthermore, a simple mediation model considering, for instance, telework as a predictor of work engagement via satisfaction of autonomy needs is significant (indirect effect: 0.18, SE = 0.06, IC 95% [0.06, 0.31]) or predicting well-being (indirect effect: 0.14, SE = 0.05, IC 95% [0.05, 0.25]). The same pattern occurs for the practice of taking the pet to work (work engagement: indirect effect: 0.15, SE = 0.07, IC 95% [0.01, 0.29]; well-being: indirect effect: 0.12, SE = 0.06, IC 95% [0.01, 0.24]). Thus, pet-friendly practices that are related to being near the pet while working (either by teleworking or taking the pet to work) also appear to satisfy the need for autonomy among employees which, in turn, is associated with increased levels of feeling vigorous, being dedicated and immersed on the work tasks, and at the same time increased well-being levels. Some studies have already reported consistent findings [40]. For instance, in a daily diary study, Junça-Silva [22] evidenced that pet owners who were working from home and had the opportunity to interact with their pets during the working day had increased levels of both work engagement and performance when compared to the days in which they were working far from their pets (i.e., at the office). Furthermore, Sousa et al. [8] in an experimental study showed that the presence of pets increased the perception of social responsibility and employee organizational commitment. Hence, pet-friendly practices that resort to the presence of human-animal interactions potentially satisfy the need for autonomy leading to increased levels of work engagement and well-being.

RETRACTED

Additionally, pet-friendly practices positively influence work engagement and well-being through the satisfaction of both competence and relatedness needs. For instance, when working remotely or when employees who own pets take these to work, they may benefit from working nearby them; further, they do not have to be worried about their pets being home alone for long hours which makes them more focused on the work, and feeling more competent and confident, and in turn makes employees engaged and happier [73]. Other studies have shown that employees who are not worried about pets being at home all day unsupervised experience less stress [4]. Studies have shown that stress is higher in those who do not own a pet [36]. Concerning productivity, allowing pets to be at work (such as in the case of remote work or workplace facilities) can also increase productivity, as employees may miss fewer sick days, adding the fact that they are accompanied by their furry friend [24], performing better without the stress of worrying about them at home [11, 48].

From a social exchange perspective, it is likely that by being allowed to work from home, pet owners feel a sense of duty and gratitude to their organization, which consequently can lead to positive outcomes, such as feeling vigorous, dedicated, and absorbed in work [12, 13]. Further, working in an organization with pet-friendly practices –not only including telework or taking the pet to work but also other pet-friendly practices, such as having a pet-friendly culture or having the day to take the pet to the veterinary, among others – that share similar values with employees will likely to make these more connected to the organization and satisfying their need for relatedness which, in turn, may create happy and engaged employees. For instance, Grandin and Johnson [74] stated that the “strong psychological and emotional attachment to, together with the positive interactions with animals, form a special bond that improves human quality of life—emotionally, psychologically, physically, and spiritually” (p. 22). In this line, some studies have shown that pet ownership, human-animal interactions, and the human-animal bond have social and individual benefits [3, 8]. In terms of physical and psychological health, studies demonstrated that pet owners have a reduced risk of cardiovascular disease and fewer sick days [13]. Pets’ behaviors dispel laughter, promote humor and entertainment, reduce depression, and contribute to long-term well-being [75]. Pet ownership also provides social support since they are conceptualized as emotional therapists [27]. The support received from pets can encourage humans to have more social interactions with other humans, such as their work colleagues [76]. Beyond this, Barker [45] supported that pet-friendly workplaces are indicators that organizations value and worry about their employees’ well-being. Furthermore, when an employee needs to choose between a pet-friendly organization and a traditional one, candidates (with pet-friendly values or with pets) tend to choose the first [33, 42].

RETRACTED

In conclusion, there is a pressing need for clarity regarding pet-friendly practices, as many managers seem to narrow their scope solely to allowing pets in the workplace, overlooking the broader spectrum of potential benefits, such as enhanced well-being. Moreover, it's crucial to recognize that pet-friendly initiatives significantly impact both well-being and work engagement by fulfilling employees' fundamental needs for relatedness and competence.

### Practical implications

As time goes by, the interest of organizations in being pet-friendly workplaces tends to increase and it is, therefore, important to provide recommendations to human resources managers. This study contributes to this direction.

First, from the managers' perspective, the findings show that although they are familiar with the topic, there are still doubts and uncertainties about pet-friendly practices and their potential benefits. Their main assumption is that pet-friendly practices are limited to taking the pet to the workplace, although they believe that they can contribute positively to productivity and work engagement, and reduce stress and anxiety [1, 5, 18]. Plus, these measures must be implemented gradually since Portugal has a conservative culture with a closed mind toward new issues and practices.

Although there are benefits, there are also some limitations and disadvantages related to pet-friendly practices. Firstly, the financial budget of each organization has to be considered, as these measures require an initial investment that will impact financial management. Although there is a possible long-term return (in terms of productivity and reduced absenteeism and turnover), organizations must be financially stable to implement all the measures strategically and progressively. Moreover, it is essential to consider the perspective of all employees when thinking about implementing new measures to avoid the opposite effect.

There are different forms of pet-friendly practices, and organizations can implement them from simpler to more complex ones. Organizations that are hesitant to become pet-friendly should start with simple measures and gradually adopt more complex ones. The main concern is to consider the needs of the workplace and employees. Not all pet-friendly practices are aimed at bringing the pet to the workplace. For instance, organizations can implement different pet-friendly measures, from simple options to more complex actions. Simple measures include offering employees vouchers for pet services, veterinary health care coverage, such as pet insurance, or work flexibility (such as remote work). Some organizations, such as Confirm BioSciences, Nestlé, and Fidelidade give employees flexibility (e.g., remote work) to attend to their pet’s needs during the workday by granting flexible work arrangements to work nearby their pets [5]. For example, flextime is helpful for employees with pets who may need a flexible working schedule to check on their pets or walk them during the day [6–8].

RETRACTED

Another option is pet bereavement days in case employees need to bereave a pet's death. There are however more challenging options to implement, including for instance, allowing the opportunity for employees to bring their pets to work and offering on-site perks such as walking services, pet daycare, outdoor enclosures, and grooming services [42]. The implementation of these measures is expected to be gradual.

A more complex option of pet-friendly practices includes the opportunity to take an employee’s pet to work. This practice, although complex in terms of physical facilities, is particularly beneficial for employees who do not need to be concerned about their pets being home alone for long hours. This trend seems to be on the rise with a small but growing number of employers that allow pets in the workplace [9, 10]. Organizations such as Amazon, Autodesk, Ben Jerry’s, Nestlé Purina, P&G Pet Care, and Zynga, among others, regularly allow their employees to bring their pets to work. Allergies and phobias are also important limitations in the case of the practice of taking pets to the workplace.

The next recommendation for policymakers is to include their employees in the implementation process as these measures can have an unequal effect on people who do not have pets, and this is a factor that should be considered in the early stages of the process. For instance, it is necessary to conduct employee surveys or even hold meetings with everyone to discuss the topic and analyze everyone's perspective. Organizations should frequently check employees' attitudes toward existing policies regarding pets to ensure fair treatment for all. Organizations may need to reassess their pet-friendly approach when hiring new employees to make sure that they fit with the culture and values. To improve employee performance and, consequently, organizational productivity, employers should promote both individual and healthier work environments, and pet-friendly practices are one example of measures that can be implemented in this direction.

RETRACTED

Pet-friendly practices should be formally and regularly evaluated to determine the success of the initiative, provide evidence of their impact, and improve the program so that future efforts are implemented more effectively. It can be helpful to compare the policies and procedures of similar organizations that have successfully instituted pet-friendly cultures.

### Limitations and future research directions

First, regarding the second study, the use of self-reported measures together with a two-wave design may have created the common method bias [63]. However, some procedures (such as the different confirmatory factor analysis, the reliability analysis, and Harman’s single factor analysis) show that the common method bias is not a severe issue in the study. Yet, the study relies on a two-wave design which may create some bias in the interpretation of the results as, for instance, well-being and work engagement appear to fluctuate over time [40]; thereby, future studies should consider alternative designs, such as daily diary studies, to test the model. Another limitation is related to the sample composition. In the second study, 95% of the participants were women which poses a limitation to the generalizability of the findings. Hence, future studies should test the model with a more homogeneous sample. At last, the use of a single-country factor is a significant limitation impacting the study's generalizability. Therefore, future studies could explore and test the model in different countries.

Future studies should continue to investigate the impact that pet-friendly practices have on employee well-being and at organizational levels observing their long-term effects. Experimental studies are essential. For instance, implementing these practices in organizations to verify their effects on the organization, and evaluating the differences in terms of satisfaction, productivity, well-being, motivation, and stress reduction should be developed.

It is still important to explore the disadvantages of the practices and possible practical solutions to them. As it is still an embryonic issue, research should be further explored to provide all the information for designing practical recommendations for organizations.

## Conclusions

In an evolving landscape, organizations are increasingly exploring novel methods to attract and retain talent, prioritizing employee engagement, performance enhancement, and job satisfaction. This study underscores the significance of pets in people's lives, acknowledging them as integral family members that bolster overall well-being. Consequently, embracing pet-friendly initiatives offers a plethora of benefits over drawbacks, urging organizations to invest in flexible work arrangements, financial subsidies encompassing veterinary care, accommodation, and pet insurance, alongside initiatives such as adopting a pet mascot or instituting designated 'pet-days'. These measures not only elevate well-being but also foster heightened work engagement, thereby motivating their workforce.

RETRACTED

Portugal’s relative unfamiliarity with this concept stems from societal conservatism and a dearth of discourse, both informally and in business circles. Additionally, financial considerations weigh heavily on the adoption of such strategies. Furthermore, managerial impartiality is crucial given the varied organizational responses to pet-friendly policies, necessitating a meticulously planned implementation strategy to avert perceptions of inequality among employees. However, it's apparent that both managers and employees possess limited insight into the breadth of pet-friendly practices, often conflating it solely with allowing pets in the workplace. Hence, there's a pressing need for awareness campaigns and open discussions to elucidate the array of viable initiatives, prioritizing simpler strategies before delving into more intricate ones like allowing pets in workplaces.

The study delves into the potential impact of pet-friendly practices on employee well-being, particularly in fulfilling psychological needs. It reveals a tangible correlation between such initiatives and heightened well-being and work engagement, underscoring their role in fulfilling employees' needs for competence and social connection.

Ultimately, pet-friendly policies emerge as pivotal facets of employees' lives. As further research continues to spotlight their manifold benefits, organizations will increasingly recognize the value of integrating these practices into their operational frameworks, bolstering confidence in initiating the implementation process.

## Data Availability

Data will be made available upon reasonable request on the corresponding author.
